This article has been retracted.

# The Data Analytics of Finance Impact on the Rural Development Combining Financial Constraint and Economic Growth Theory

**DOI:** 10.1155/2022/9989076

**Published:** 2022-04-20

**Authors:** Xiaoxiao Guo

**Affiliations:** College of Commercial, Wuxi Taihu University, Wuxi 214064, Jiangsu, China

## Abstract

In order to solve the predicament of rural economic development, China's rural areas have spontaneously formed a rural financial system with rural characteristics. With the deepening reform of rural finance, Rural Commercial Bank was restructured on the basis of rural credit cooperatives in the past. It can be said that Rural Commercial Bank is a rural financial institution born in rural areas. Therefore, the development of the local rural commercial bank and the development of the local rural economy have been integrated, and the core force in rural finance is the Rural Commercial Bank. It is precisely because of the core position of China's rural commercial banks in rural, when Chinese scholars conduct research on rural finance, they often choose rural commercial banks as the research object. Based on this, when the article studies the impact of rural finance on the rural economy, it also chooses rural commercial banks as the research object. Finance that the rural commercial banks are used as the starting point to carry out the research work on their local rural finance. This article takes D County Rural Commercial Bank as an example to introduce and analyze the development status and development process of D county's rural finance. Using the method of empirical research, this paper studies the impact of the development of agricultural-related business of rural commercial banks on the rural economy. In addition, according to the empirical research results, a set of financial innovation countermeasures to promote rural economic development is proposed. Through the research on the influence of rural financial institutions in D county on the rural economy, it can be seen that providing new directions and new methods for the development of China's rural economy from the perspective of finance. It provides a reference for promoting the stable and effective development of the domestic rural economy. The survey shows that rural deposits have maintained a rapid upward trend. The total amount increased rapidly from 2.219 billion yuan in 2012 to 6.039 billion yuan in 2018, with an average annual increase of 637 million yuan.

## 1. Introduction

In order to solve the predicament of rural economic development, China's rural areas have spontaneously formed a rural financial system with rural characteristics. With the deepening reform of rural finance, the rural commercial bank was restructured on the basis of the rural credit cooperatives in the past. It can be said that the rural commercial bank is a rural financial institution born in the countryside. It is located in the deep economic development of the province and the vast rural areas, with the help of China's three existing urbanization strategies. With the goal of poverty alleviation and rural revitalization, it will promote the province's economic development and the transformation of rural and private economies. Like decades of economic growth, rural commercial banks and their successors have grown with the development of the rural economy. As a result, the development of local rural commercial banks is integrated with the local rural economy. The core driving force of rural finance is rural commercial banks; it is precisely because of the core position of rural commercial banks in rural finance that Chinese scholars often choose rural commercial banks as the research object when conducting research on rural finance. Based on this, when the article studies the impact of rural finance on the rural economy, it also chooses rural commercial banks as the research object and takes the rural commercial bank as the research starting point to carry out the research work on its local rural finance.

Since the financial development theory was put forward, many economic researchers have begun to explore the relationship between financial development and economic growth and pointed out that financial development must abide by the principle of moderation. The backward financial development will have a negative impact on economic growth. In the mid-1980s and 1990s, debt and financial crises began to appear in developing countries, and in 2008, there was also a financial crisis, so people's attention to the relevant theories has been deepened, thus prompting people to pay more attention to the relationship between financial development and economic growth. Financial development is regarded as the main factor of economic growth, and rural finance has played an important role in rural economic development. Rural finance can bring an important source of funds to rural economic development, and it is also the most important part of modern finance. Therefore, the continuous increase in the theoretical exploration of rural finance and economy has important theoretical significance for the study of the development of rural economy and the increase of farmers' income.

The article combines the theory of financial constraints, Patrick's theory, economic growth theory to analyze the different development stages of D county. At the same time, it conducts empirical research on the rural finance of D county by constructing the relation model between rural finance and rural economy represented by rural commercial banks and further studies the role of rural finance on rural economy. Most of the existing literature analyzes the relationship between financial development and rural economic growth. There are still relatively few studies on the relationship between rural finance and economic growth represented by rural commercial banks. Previous studies have mainly studied the relationship between rural finance and economic growth from the perspective of a country or a large region, and few people have conducted in-depth research based on a county. This paper mainly studies the rural financial innovation and rural economic growth in D county based on the county level.

## 2. Related Work

Experts at home and abroad have also conducted many studies on Internet big data and rural economy. Yu et al. believes that China's rural cooperative financial organizations have played an important role in dispersing agricultural production risks, increasing farmers' income, and stimulating the overall development of the rural economy [1]. Zhou et al. presents several applications including smart grid, smart transportation, and smart city to demonstrate how IOT based on fuzzy/edge computing can be implemented in real-world applications [2]. In order to reduce the amount of data collected by the Internet of Things and improve the processing speed of big data, Xue proposed a method of compressed sensing sampling. Aiming at the high computational complexity of the compressed sensing algorithm, the multiobjective optimization particle swarm optimization algorithm is used to improve the search terms of the gradient projection sparse reconstruction algorithm (GPSR-BB) [3]. Mostafa et al. believes that wearable devices and mobile applications are now effectively integrated with telemedicine and telemedicine to build the medical Internet of Things [4]. Shi pointed out that the optimization of industrial structure is an important explanatory variable for economic growth, and the allocation of production factors among industries affects the evolution of industrial structure and thus affects economic growth [5]. Yang Y has done a lot of research work to deal with these problems and find a better way to eliminate these risks in order to protect IOT devices or at least minimize their impact on user privacy and security requirements [6]. These studies provide a lot of evidence for these experiments, but due to the short study time, there are some doubts about the tested samples, which makes the test results need to be confirmed by everyone.

## 3. Advanced ICT in the Internet of Things

The Internet of Things is an important part of the new generation of information technology. As the name suggests, “The Internet of Things is the Internet of things connected.” The core and foundation of the Internet of Things is still the Internet, an extended network based on the Internet. At present, the definition of the Internet of Things can refer to the relevant literature. Therefore, the Internet of Things is to connect any item with the Internet through radio frequency identification (RFID), infrared sensors, global positioning systems, laser scanners, and other information sensing equipment, according to the agreed protocol, to exchange and communicate information to achieve a network for intelligent identification, location, tracking, monitoring, and management of items. Embedded intelligence in objects can enhance the power of networks by transferring information processing capabilities across the network boundaries. Finally, the advantages of miniaturization technology and nanometers mean that increasingly smaller objects can interact and connect. All these technologies come together to form the Internet of Things, connecting objects in the world sensory and intelligently. At this stage, the concept of the Internet of Things has a new statement: the Internet of Things is to combine various information sensing devices with the Internet to form a huge network, so that all items are connected to the network for easy identification, management, and monitoring. On the basis of the integration of the application and ultimately provide people with ubiquitous all-round services, Figure 1 shows ITU-T research on the Internet of Things.

Object-embedded intelligence enhances the capabilities of networks by transmitting information processing capabilities across network boundaries. The advantages of miniaturization and nanotechnology mean that even smaller objects can interact and connect. All these technologies combine to form the Internet of Things, which connects sensual and intelligent things to the world [7]. So far, the concept of the Internet of Things has a new release: the Internet of Things is to integrate different Internet information monitoring devices into a large network so that everything is connected to the Internet, which is easy to identify, manage, and monitor and provide universal services. Figure 1 shows the ITU-T research on the Internet of Things.

In order to be able to connect physical and virtual objects to provide better services, IOT needs to leverage a range of existing and/or evolving advanced technologies such as machine-to-machine communication (M2M), data mining and decision making, self-organizing networking, security and privacy protection, cloud computing, and sensing and triggering technologies. The reference model of the Internet of Things is briefly summarized, as shown in Figure 2 [8].

### 3.1. Data Acquisition Protocol

In order to establish appropriate channels to obtain data from edge devices, although there is no consistent protocol to support data collection, corresponding mechanisms have emerged in some specific fields. Of course, it is necessary to accept a protocol for devices to communicate with each other, and a cloud that can perform aggregated analysis is necessary. Some companies are taking a dedicated route, while others are affected by open source. Likewise, other concerted efforts to bring about more IOT standardization have emerged, including the Open Interconnection Consortium (OIC), the AllSeen Alliance, the Thread Group, the Industrial Networking Consortium (IIC), and IEEEP2413. Developing an open source ecosystem has its advantages as more influential communities can be formed. Moreover, taking into account the participation of user groups in development and data collection, the development becomes relatively easy and extensive. Since these devices collect high-dimensional and capture high-frequency device states, this will in turn require the support of high-bandwidth connections. In addition to the OIC, AllSeen, llC, and IEEEP2413 introduced in the article, there are many other standardization organizations engaged in the research and formulation of standardization related to the Internet of Things.  Figure 3 gives the relevant standardization organizations and their general scope of study [9].

### 3.2. Transmission Mechanism of Rural Finance to Rural Economic Growth

Letting the total output of the rural economy be *Y*, *C* is the total rural consumption, *S* is the total rural savings, *I* is the total rural investment, and *t* is the time. Since the agricultural production sector produces only one product, one part is used for consumption and the other part is used for savings. Moreover, the total rural savings can be completely transformed into the total rural investment, so the basic total balance equation of the rural economic sector is:

(1) $$\begin{array}{c} Y\left(t\right)=C\left(t\right)+S\left(t\right). \end{array}$$

Having:

(2) $$\begin{array}{c} Y\left(t\right)=C\left(t\right)+I\left(t\right). \end{array}$$

Available:

(3) $$\begin{array}{c} S\left(t\right)=I\left(t\right). \end{array}$$

The total social capital stock is equal to:

(4) $$\begin{array}{c} K\left(t+1\right)=K\left(t\right)+I\left(t\right). \end{array}$$

Letting the depreciation rate of the capital stock is *β*, then the stock is equal to:

(5) $$\begin{array}{c} K\left(t+1\right)=\left(1-\beta \right)K\left(t\right)+I\left(t\right). \end{array}$$

Then the savings rate is:

(6) $$\begin{array}{c} s=\frac{S\left(t\right)}{Y\left(t\right)}. \end{array}$$

The output capital rate is:

(7) $$\begin{array}{c} \lambda =\frac{Y\left(t\right)}{K\left(t\right)}. \end{array}$$

The joint formula is:

(8) $$\begin{array}{c} K\left(t+1\right)=\left(1-\beta \right)K\left(t\right)+S\left(t\right). \end{array}$$

Substituting expressions include:

(9) $$\begin{array}{c} \frac{Y\left(t+1\right)}{\lambda }=\frac{\left(1-\beta \right)*Y\left(t\right)}{\lambda +sY\left(t\right)},\\ w+\beta =s\lambda . \end{array}$$

Substituting into:

(10) $$\begin{array}{c} s\left(\frac{\Delta Y}{Y,\eta }\right)\lambda =w+\beta . \end{array}$$

Taking the rural finance and rural economy under closed conditions as the object, it can be assumed that the total output of the rural economy is a linear function of the capital stock. It is assumed that the marginal product efficiency of capital is increasing, thus introducing financial factors. Letting the total rural output be *Y*, the marginal product efficiency of capital be *A*, and the capital stock be *K* [10].

(11) $$\begin{array}{c} Yt=AKt,\\ It=Kt+1-Kt,\\ It=Kt+1-\left(1-\beta \right)Kt. \end{array}$$

Since the economic growth rate of *t* + 1 can be expressed as:

(12) $$\begin{array}{c} t+1=\frac{\left(Yt+1-Yt\right)}{yt}. \end{array}$$

The substitution formula is:

(13) $$\begin{array}{c} wt+1=\frac{\left[It+\left(1-\beta \right)Kt\right]}{Kt}-1\\ =\frac{It}{Kt+\left(1-\beta \right)}-1\\ =\frac{A*It}{Yt-\beta },\\ w=A\left(\frac{I}{Y}\right)-\beta . \end{array}$$

### 3.3. Model Running Result Verification

The running effect of the model can be checked by comparing the relative error between the results of the model running and the actual data. It is generally believed that the relative error of each variable is less than 10%, and the prediction performance of the model can be judged better. The level of rural financial development is one of the key indicators of the rural financial system, and the chart below is its prediction result. It can be seen that the error of the level of rural financial development is controlled within ±10%, and it can be considered that the model prediction effect is good, as shown in Figure 4 [11].

Table 1 is a fitting table of the rural financial development level. The rural financial development subsystem mainly includes four first-level indicators: the overall level of rural financial development, the structure of rural financial deposits and loans, the structure of interest rates, and the level of development of rural financial institutions. Since the rural financial deposit and loan structure and interest rate structure reflect the status of rural financial institutions, rather than an absolute indicator, it is impossible to directly see the development trend from the results of system operation. Here, mainly examining the development level of rural finance and the development level of rural financial institutions [12]. Using Vensim to analyze the model, the operation results of the main indicators of the rural financial development subsystem are presented in Figure 5 and Table 2:

## 4. Influence of D County Rural Finance on Rural Economy

The article focuses on the development status of rural commercial bank finance and rural economy in D county. The study found that the Rural Commercial Bank of D county occupies the first place in the county's rural finance at this stage and is in an absolute leading position. The article mainly based on the operation data of D County Rural Commercial Bank, and at the same time, temporarily replaced the rural financial development indicators with rural deposits and loans and rural fixed asset investment, to construct relevant models for empirical analysis. Therefore, when exploring the relationship between rural finance and rural economy, the research on rural commercial banks has become the top priority. After analyzing several independent variable indicators that affect the rural economy of D county, the analysis results are further extended to the impact of D county's overall rural finance on the rural economy for discussion and analysis [13].

### 4.1. Construction of Indicator System

The reason why the rural deposit and loan indicators of rural commercial banks are used as an alternative indicator of the development of rural finance is to take into account the actual situation of rural finance in county D: D County Rural Commercial Banks are the main part of D county rural financial institutions, accounting for 61.2% of the total number of D county rural banks. Rural deposits accounted for 53.88% of the total rural deposits in county D, and 85.5% of the total agricultural loans in county D. At the same time, the development of the financial market in the rural areas of D county is still relatively slow. Rural deposits and loans are the most direct manifestation of rural financial activities, which can intuitively show the impact of various financial policies on the economy. The main financial activities in the rural areas are still dominated by the credit of rural commercial banks, so this article chooses rural deposits and loans of rural commercial banks as one of the financial development indicators. As for the selection of fixed asset investment as one of the indicators, it is considered that it represents the power source of rural economic development in D county to a certain extent.

In order to overcome the heteroscedasticity of the data selected in this paper, the paper takes the natural per capita income of rural areas (RJSR), rural commercial bank deposits (NYCK), rural commercial bank rural loans (NYDK), and fixed assets (GDZC) in D county. The logarithm is used as a variable for empirical analysis, which is represented by DXRJSR, DXNYCK, DXNYDK, and DXGDZC in turn [14].

### 4.2. Data Sources

The sample interval selected for the empirical analysis of the article is from 1998 to 2018, and the data comes from the financial statements and internal journals of D County Rural Commercial Bank in the calendar years from 1998 to 2018 and the “D county Statistical Yearbook” over the years. Apart from the description, the data were not processed otherwise. The article will use EViews measurement software to process and test relevant data, as presented in Table 3 [15].

Here, using the more commonly used Fuller (ADF) unit root test method, and the predecessor of the Fuller test is the DF test. The DF test is often used to detect the nonstationarity of variables. As for the practical series of unit roots, this time series is actually relatively nonstationary. Using EViews software to test the variables in the article, the per capita income of rural areas in county D, rural loans, rural deposits, and the unit root of fixed asset investment, the test results are presented in Table 4:

A short-term dynamic relationship is established, that is, the error correction equation. The variables in the long-term relationship model are reconstructed in the form of first-order differences, and the residual sequence generated by the long-term relationship model is introduced as an explanatory variable. Test, insignificant items are eliminated one by one, until the final expression method is found.

If there is a cointegration relationship between *y* and *x*, estimating the cointegration regression equation and calculating the residual sequence *et*:

(14) $$\begin{array}{c} yt=\alpha +\beta x_{t}+\varepsilon_{t},\\ et=yt-\overset{⌢}{\alpha }-{\overset{⌢}{\beta }}_{0}x_{t}. \end{array}$$

Using *et* − 1 as an explanatory variable, estimating the error correction model:

(15) $$\begin{array}{c} \Delta y_{t}=\alpha +\beta_{o}\Delta x_{t}+\gamma e_{t-1}+v_{t}. \end{array}$$

### 4.3. Overall Development of Rural Economy in D County

In the past two years, due to the influence of macro factors, its growth rate has slowed down and the agricultural development in the region has also been greatly affected. In 2017 and 2018, after the rural economy was affected by price factors, its growth rate was 4.2% and 0.83%, respectively. Compared with previous years, the rate of increase has shown a significant downward trend, as presented in Table 5 [16].

As can be seen from the table, in the past ten years of development, the growth value of the primary industry in the region has always maintained a relatively high growth trend and subject to the influence of external macro factors; the growth rate has declined in 2017 and 2018. As far as the growth value of the primary industry is concerned, its share in the region's total economic output has maintained a downward trend every year, which is consistent with the requirements of the domestic urbanization policy. In addition, in terms of total volume, the primary industry has shown a continuous upward trend. In 2000, its increase value was 185 million yuan, and by 2018, it had increased to 3.905 billion yuan, the average annual growth rate has reached 18%, which is larger than the domestic average growth rate. The detailed growth trend from 2000 to 2018 is as shown in Figure 6 [17].

After the reform and opening up, the national economy has achieved rapid development, and the income level has also been significantly improved. The economic development goal of providing food and clothing at the beginning has continued to rise. The per capita disposable income of households in rural areas has risen rapidly, and by the end of 2017, the living standards of farmers in the region had already achieved a moderately prosperous level. Its urban per capita disposable income reached 17,387 yuan, a year-on-year increase of 8.9%; the per capita consumption expenditure of urban residents was 13,658 yuan. The per capita disposable income of rural residents was 8,726 yuan, an increase of 8.8%, of which wage income was 2,101 yuan, net operating income was 4,506 yuan, net property income was 286 yuan, and net transfer income was 1,833 yuan; the total per capita living consumption of farmers was 6,218 yuan. In the past ten years, although income has risen sharply, it can also be concluded that there is a large gap between the per capita disposable income of urban and rural residents in the region, which also causes the loss of labor in the region. Coupled with the continuous development of urbanization, the demand for labor in urban areas has continued to increase, and a large number of rural people have begun to pour into cities and towns. A large number of laborers began to abandon agricultural production and poured into cities to work. In 2014, the region gave a three-year development goal of major changes and accelerated the pace of urbanization. First of all, the number of employment in the primary industry has been continuously reduced, which has achieved great results in terms of urbanization, but it has brought a huge impact on the economic development of rural areas. However, there has been a wide range of declines in both employment and absolute numbers, as shown in Figure 7 [18].

It can be seen from Figure 7 that in county D, the per capita income of urban residents has grown rapidly. Especially in recent years, revenue has continued to grow and the growth rate is also very large. The disposable income of urban households increased from 5,000 yuan in 1997 to 35,000 yuan in 2017, an increase of nearly seven times. Correspondingly, although the growth rate of the per capita income of rural households in D county is also increasing, it is very slow compared with the per capita income of urban areas, and the per capita income increased from 603.5 yuan in 1997 to 8,726 yuan in 2017. At the same time, it can be seen from the income gap ratio that since 2010, the growth rate of rural per capita economic income has gradually increased with that of urban economic income, and there is still an increasing trend. In 2006, the total number of primary industry personnel in the region was 161,200. According to relevant data, by the end of 2016, the total number of personnel had decreased to 82,700. In 2006, the total number of employed persons in the primary industry accounted for 39.6% of the total employment; by the end of 2016, the number had decreased to 26.9%. The main factor leading to this situation is that the advancement of science and technology has caused the demand for the total number of personnel in agricultural production to begin to decrease, but the most critical factor is the loss of personnel caused by external demand. In some rural families, only the elderly and children are left behind, and most of the laborers who can carry out agricultural production choose to go out, which causes a large number of farmland to be abandoned and directly affects the development of agriculture in the region [19].

Affected by factors such as geography, land and climate, agricultural production, and economy have always suffered a very serious impact. Because of the continuous development of modern technology and the substantial improvement of production levels, many production problems have been solved. Rural economic development has also begun to focus on the labor force at the beginning to the current technology-based development. The demands on machinery and technology are constantly increasing, so the dependence of agriculture and rural development on technology is beginning to increase. The main factor affecting its technological and mechanized production is the input of farmers' fixed assets. This type of input can be further divided into fixed asset input of rural farmers and nonagricultural households. The former refers to the value of fixed assets such as housing buildings and mechanical facilities. The latter refers to construction projects with a planned total investment of more than 380,000 yuan carried out by registered enterprises, institutions, and administrative agencies. In 2000, the total investment in fixed assets of rural households in this area was 1.866 billion yuan, which reached its peak in 2011 and increased to 3.528 billion yuan, followed by a corresponding decrease, and by the end of 2018, it was only 1.922 billion yuan [20].

### 4.4. Positive Correlation between Rural Fixed Assets and Rural Loans and Rural Economy

Among the rural deposits, rural loans, and rural fixed assets, the most obvious impact on the rural economy is rural fixed asset investment. In addition to rural fixed asset investment, rural loans have a greater impact on the rural economy, and capital turnover and easy loans can facilitate better investment in the rural economy.

1. The impact of rural financial fixed assets to analyze the investment in rural financial fixed assets is generally shown. At the micro level, it is an effective improvement of the efficiency of rural financial services. At the macro level, it is the growth of the loan-to-deposit ratio. The improvement of service efficiency is due to the continuous reduction of service costs with the investment of rural financial fixed assets. The main features of finance in this region are that “the number of transactions is relatively large, the scale is small, and the coverage area is relatively broad,” which also causes the service cost of financial institutions in the region to be relatively large, and when the service efficiency in the region continues to improve, the application of various information technology, the service cost has been greatly reduced. The establishment of the Hewlett Packard enterprise rural financial payment and settlement system includes the continuous improvement of bank account and bank card services in rural areas, the continued growth of outlets of financial units in the region, and the rapid development of new forms of payment. The establishment of the rural financial payment and settlement system in county D has led to a reduction in the corresponding service costs. By the end of 2012, there were 2.36 billion personal accounts created by financial institutions in rural areas in China, and 1.35 billion bank cards were issued in total. The number of rural financial units interconnected with the central bank's payment system is more than 70,000, covering 60% of the area, which also effectively improves the payment and settlement efficiency of rural financial units. In addition, with the continuous development and application of information technology, the mobile and online payment of rural finance has achieved rapid development, and the comprehensive development of third-party payment services has effectively improved the service efficiency of financial units and reduced their costs. As of June 2018, Rural Commercial Banks (Rural Credit Cooperatives), Agricultural Banks, and Postal Savings have established 829,000 cash withdrawal outlets in rural areas, covering 85% of administrative villages. This is also the manifestation of “demand following” in Patrick's theory. The final result of the development of rural finance is to support the development of the rural real economy [21].
2. Analysis of the impact of rural loans from 2012 to 2018, financial institutions in the region have always increased their lending to agriculture, and their proportion in total loans has also increased significantly compared with before. With the increase in the amount of social loans, agricultural investment and rural infrastructure construction have been greatly improved, which greatly promoted the growth of the rural economy. Its data support mainly comes from the internal data and network data of financial institutions in D county. From 2012 to 2018, the amount of agriculture-related loans provided by D County Rural Commercial Bank is shown in Figure 8 [22].

Figure 8 shows the amount of agriculture-related loans provided by D County Rural Commercial Bank from 2012 to 2018. The amount of agriculture-related loans has increased every year, from 1.36 billion yuan in 2012 to 2.521 billion yuan in 2018. This reflects the way in which “supply leadership” develops in Patrick's theory. The most important financial supply is the supply of funds, including the loose monetary policy of the central government, which is the main factor that promotes the growth of various demands in rural areas. At the same time, it is also a direct reflection of the impact of rural finance on the rural economy, thereby realizing the further development of the rural economy [23].

Among them, only rural deposits are negatively correlated with rural economic growth, that is, the more rural deposits in a fixed period, the poorer the rural economy is. Because the increase in rural deposits will allow agricultural funds to flow into rural financial institutions, and under the current system, most of China's rural financial institutions will use this part of the funds in lending to economically developed areas or handing over to the central bank, agreement deposits, etc., all of which have formed a “blood-drawing effect” on the financial market in rural areas; to a certain extent, it hindered the development of the local economy and rural deposits are also closely related to the country's macroeconomic policies. In order to stimulate consumption and encourage investment, the state will implement a lower benchmark deposit rate, which will give people more reasons to invest funds instead of storing them in banks. So as to achieve the purpose of accelerating economic growth, the increase in the scale of rural financial development is generally reflected in the growth of the total number of rural financial intermediaries and the growth of total financial assets. Since the reform and opening up, the economy of rural areas has achieved rapid development, which has led to a significant increase in farmers' income, which has provided an important basis for the growth of rural savings. With the help of the research, it can be concluded that during the recovery period of the rural financial system, it also showed an important saving effect. Rural deposits maintained a rapid upward trend. The total amount increased rapidly from 2.219 billion yuan in 2012 to 6.039 billion yuan in 2018, with an average annual increase of 637 million yuan. In particular, D County Rural Commercial Bank, after the comprehensive reform, agricultural-related loans increased from 1.368 billion yuan in 2012 to 2.521 billion yuan in 2018, with an average annual increase of 192 million yuan. Its rural deposits increased from 1.42 billion yuan in 2012 to 3.254 billion yuan in 2018, with an average annual growth of 306 million yuan, as shown in Figure 9 [24].

From the research, it can be concluded that the total number of rural loan balances and the rising rate in D county have maintained a rising trend, which brought an important financial guarantee to the economic development of the region and promoted its development. In theory, this will help bring important capital accumulation to the rural economic development of D County, and the total investment in fixed assets will continue to rise, and the proportion of rural GDP will continue to grow. At the same time, this will also contribute to the continuous improvement of rural consumption levels, the continuous expansion of industries, and the continued growth and development of township and village enterprises, which in turn contributes to further economic development in rural areas. One aspect that needs to be explained here is that the negative correlation between rural deposits and rural economic growth is based on a fixed period of time, that is, the total amount of rural deposits is constant. If the proportion of rural financial institutions in rural deposits is higher, it will negatively affect the development of rural economy. However, by combining the data in Figure 9 with the Harold–Dormer equation in the economic growth theory, I can still conclude that an increase in the savings rate can promote an increase in the economic growth rate. However, its impact factor is still achieved by increasing the amount of loans. Because banks have a control over the loan-to-deposit ratio, which determines the level of operating efficiency, banks will increase the amount of loans correspondingly after the increase in deposits, thereby promoting the development of the rural economy.

In terms of the distribution of large and medium-sized commercial banks, many commercial banks are established in D county towns with relatively good economic development, and only a few branches are established in rural areas. In terms of business, the five major domestic commercial banks, whose main service entities are also large and medium-sized enterprises in the region and rural areas, have relatively good returns. Small and medium-sized enterprises of a certain size, specifically in terms of small enterprises, do not give much help, letting alone the production of farmers. Financial institutions have not fully demonstrated their own policy and financial functions nor have they brought comprehensive services to “agriculture, rural areas, and farmers.” As far as the rural credit cooperatives, which are the main force supporting agriculture, have lost the main attribute of cooperative finance, their commercial operation mode makes their supporting agriculture power significantly insufficient, as shown in Figure 10.

As shown in Figure 10, whether it is a new type of financial institution or a large and medium-sized commercial bank in the proportion of loans in various industries, large enterprises and small enterprises are the main force of loans in D county. This situation has seriously hindered the growth of the rural economy in D county. A single type of loan, lack of innovation, and lack of agricultural insurance make it difficult to obtain loans, although the credit fund has increased, it cannot meet the demand and speed of farmers and enterprises. In addition, coupled with the limited loan amount for farmers and enterprises, it has also curbed the development of the rural economy to a large extent. In terms of loan business, more than 80% of farmers believe that the current interest rate cannot meet their production needs. At present, most of the rural loans in this area are mainly short-term and small loans, but in terms of the characteristics of agricultural production, only medium and long-term loans can meet the needs of their production. Every year from March to November, the agreed time for agricultural product loans is relatively short, and many farmers can only sell their crops in order to repay the loan in time, but this time the price is the lowest. There are also serious capital cycle problems in the production and operation of agriculture, aquaculture, and processing industries in the region. Short-term loans within one year simply cannot meet the requirements of agricultural production. The long term, the repayment strength of farmers, and various uncertain factors make financial units in the region unwilling to bear the corresponding risks.

## 5. Discussion

First of all, when domestic commercial banks carry out the shareholding reform, their profit characteristics begin to show. State-owned banks have begun to withdraw from rural areas, and their impact and role in rural areas is already very small. Second, as far as the agricultural development bank is concerned, its business scope and role in supporting agriculture are still very limited compared to rural financial needs. In addition, rural credit cooperatives have been developing and innovating commercial finance for more than ten years, their sense of cooperation has begun to weaken, and they will even continue to raise borrowing rates by taking advantage of their advantages in the rural market. This has led to the problem of “expensive” borrowing in the region. At the same time, Rural Commercial Bank also has many problems, such as insufficient transformation, historical factors have not been fully eliminated, and supporting facilities are relatively poor, unable to meet the current rural economy's financial needs, resulting in insufficient “three rural” services. As far as developed countries are concerned, the current agricultural development is still dominated by cooperative finance because this type of finance is not based on profit, which is consistent with the current development of agricultural economy. Finally, although China has appropriately relaxed the access requirements for the rural financial market, the access to new financial units is still not very sufficient. For example, the founder must be a bank financial unit, and the investors have relatively low shares, which results in a relatively small scale in the market, so it is difficult to show the desired effect. All in all, the domestic rural financial support for agriculture is still relatively poor, and the problems of difficult and expensive borrowing have not been effectively solved, and the supply scale of rural finance needs to be continuously expanded.

The development of rural finance in county D can effectively promote the growth of the rural economy, but it must meet the corresponding conditions so that each financial function can effectively show its own effect. The effective integration of such conditions has brought tremendous impetus to financial development and has also formed a corresponding “threshold.” The “threshold” that each region has is also different. As far as county D is concerned, the level of financial development, inflation, and education level of residents will all be possible, but the most basic one should be the level of financial development. Differences in such levels have different effects on economic development. At present, the financial development of the region has not achieved a certain level nor has it met the requirements of the “threshold,” so the function of economic growth has not been displayed. There are still many problems in the financial institution system and financial services, and there is a clear backwardness compared with the rural economy. Therefore, it is necessary to continuously promote the rapid development of rural finance and achieve continuous improvement, so as to meet the corresponding “threshold requirements.” Only in this way can rural financial and economic development achieve mutual promotion and achieve common development.

Since D county is an administrative region at the county level, it is quite different from the economic development at the provincial and municipal levels, resulting in a small number of financial institutions and a small number of large commercial banks. In order to change this form, the reform model of “cooperative finance” can be adopted. Specifically, it is necessary to build financial institutions that can be practically applied, and the original state-owned shares are gradually handed over to members to buy. The rural economy of D county has already had a foundation, and farmers generally have corresponding savings. From the perspective of policy and financial support, they are no longer the main support target. In addition, some rural credit cooperatives in rural areas focus on policy loans. Faced with this situation, commercial banks can be transformed into grassroots branches of agricultural development bank. In short, it is necessary to make the best use of the situation to choose the innovative way of commercial banks, so as to display its characteristics in the financial cooperation of the rural economy.

## 6. Conclusion

First, the article analyzes the current situation of rural finance and rural economic development in D county by combining the concepts of financial constraint theory, Patrick theory, and economic growth theory. Through the analysis, the development process of rural finance and deeply understand the mutual influence factors of rural finance in D county on the rural economy can be understood. Second, it conducts an empirical study on the influence of the financial development of rural commercial banks in D county on the rural economy. Applying the financial constraint theory, Patrick Theory, and Economic Growth Theory to the actual situation in county D to carry out an empirical study on the influence of rural commercial bank-based rural finance on the rural economy. Establishing the corresponding model according to the theory and analyzing the empirical process by selecting the corresponding indicators. It verifies the influence of the three major indicators of financial institutions' own development, deposits, loans, and related fixed assets investment on rural economic development. It is concluded that among rural deposits, rural loans, and rural fixed assets, the most obvious positive impact on rural economic growth is rural fixed asset investment, followed by rural loans. However, there is a negative correlation between rural deposits and rural economic growth in a fixed period and further extend to analyze the reasons for the problems existing in rural finance in D county at this stage. Finally, the innovative countermeasures to promote the rural economic development of D county's rural finance are put forward. The empirical conclusions of chapter four are used to verify the innovative countermeasures, and the innovative countermeasures are used to support the empirical conclusions. It has drawn innovative strategies such as developing cooperative finance, developing new loan varieties, establishing a scientific farmer rating system, improving the financial ecological environment, diversifying development, increasing policy support, and using the Internet “+”, which can effectively drive rural economic development in essence. The rural economic development of D county has a strong commonality with other rural areas in China, that is, it has developed rapidly under the drive of rural finance with rural commercial banks as the core. At present, China's rural commercial banks are in an absolute dominant position in rural finance. Therefore, the article explores the impact on the rural economy with the help of the operating data of the rural commercial banks in D county; the analysis results are still in a high degree of confidence. Letting rural finance better serve the rural areas of China and creating a rural financial structure system suitable for the domestic situation so that it can meet the development needs of domestic rural areas, serve the development of rural economy, and promote the sustainable and healthy development of China's rural economy.

## Figures and Tables

**Figure 1:** Overview of ITU-T's research on IOT standards.

**Figure 2:** Reference model for IOT.

**Figure 3:** IOT-related standardization organizations and their general scope of research.

**Figure 4:** Error rate of the rural financial development level.

**Figure 5:** Trend chart of rural financial development subsystem.

**Figure 6:** Added value of the agricultural industry in D county from 2000 to 2018.

**Figure 7:** Comparison of per capita income of urban and rural residents in county D.

**Figure 8:** D county rural commercial bank's amount of agriculture-related loans from 2012 to 2018.

**Figure 9:** Trends in rural deposits and loans and total rural deposits from 2012 to 2018.

**Figure 10:** Proportion of loans of different industries in large and medium-sized commercial banks.

**Table 1:** Fitting table of rural financial development level.

Years	2011	2012	2013	2014	2015	2016	2017	2018	2019	2020
Forecast result	66.44	58.06	67.08	71.75	71.78	75.33	76.71	76.74	76.83	77.08
Actual data	60.44	62.29	64.46	68.29	66.10	69.98	76.85	79.31	78.86	70.95
Error rate	0.00%	6.79%	4.07%	5.05%	8.59%	7.65%	−0.18%	−3.25%	−2.57%	8.65%

**Table 2:** Trend table of rural financial development subsystem.

Time (year)	Rural financial development level	Total rural amount	Farmer's cash	Farmer's deposit	Agricultural deposits	Rural GDP	Development level of rural financial institutions
2000	60.4415	25255.1	10256.9	12355.3	2642.9	41784.4	12162.5
2001	58.0608	26335.6	10416.4	12677.6	3241.57	45358.6	16494
2002	67.0836	32962.4	12413.8	15917.9	4630.73	49136.3	19393.9
2003	71.7471	38481.3	14272.1	19108.8	5100.48	53634.7	23029.1
2004	71.7772	43357.1	15722.5	22191.6	5443.1	60405.2	25467.6
2005	75.3305	51830.5	18095.3	27117	6618.27	68804.2	28053.7
2006	76.7121	57296	19531.2	29884.3	7880.42	74689.6	33349.5
2007	76.7402	60082.5	20221.7	31168.2	8692.58	78293.3	34356.7
2008	76.8292	67181.4	22001.5	35542	9637.93	87442.5	39183.3
2009	77.0809	81067.3	25655.8	44310.7	11100.7	105172	45786.9
2010	75.0234	98542.6	31299.7	52372.7	14870.2	131349	532296
2011	73.0174	114006	36643.7	60006.5	17356.1	156136	62036.5
2012	71.2845	132405	43026.9	69124.5	20254	185742	72210.5
2013	69.7934	154246	50629.2	79984.1	23632.4	221003	84051.1
2014	68.5173	180083	59646.6	92865.2	27570.8	262828	97837.8
2015	67.4341	210505	70283.6	108060	32162.1	312165	113883
2016	66.5264	246109	82739.8	125853	37514.4	369939	132500
2017	65.7813	287435	97188.6	146493	43754.1	436956	154300
2018	65.1905	334919	113747	196834	51028.1	513755	179605
2019	64.7507	388771	132430	196834	59507.9	600413	209060
2020	64.4638	448859	153102	226363	69393.4	696295	243346

**Table 3:** D county statistical yearbook.

Years	Rural per capita income (yuan)	Rural deposits of D county rural commercial bank (100 million 1 yuan)	D county rural commercial bank rural loans (100 million yuan)	Rural fixed asset investment in D county (100 million yuan)
1998	775	0.38	0.25	0.09
1999	1002	0.52	0.31	0.12
2000	1535	0.75	0.43	0.19
2001	2257	0.98	0.63	0.24
2002	2489	1.13	0.86	0.39
2003	2755	1.72	1.14	0.42
2004	2967	1.99	1.57	0.51
2005	3127	3.14	2.78	0.85
2006	3446	4.11	3.25	1.01
2007	3799	5.26	5.05	1.52
2008	3971	6.09	5.99	1.97
2009	4108	8.36	7.18	2.22
2010	4523	10.73	8.26	2.69
2011	5112	12.58	10.22	3.25
2012	6228	14.2	13.68	4.17
2013	7136	16.5	14.84	4.97
2014	7782	18.97	16.28	5.23
2015	8145	22.02	17.53	6.08
2016	8511	26.31	19.98	6.39
2017	8726	30.21	22.67	7.26
2018	8965	32.54	25.21	8.65

**Table 4:** Capital unit root test data.

Variable	Inspection form	ADF value	1% threshold	5% threshold	10% threshold	In conclusion
DXRJSR	(*c*, 0, 0)	−0.962276	−3.661661	−2.960411	−2.619160	Nonstationary
	(*c*, 0, 0)	−3.581124	−3.661616	−2.960411	−2.619160	Smooth
DXRJSR	(*c*, 0, 0)	−1.841245	−3.653718	−2.957145	−2.617434	Nonstationary
DXNYCK	(*c*, 0, 0)	−3.331645	−3.689145	−2.971815	−2.625121	Smooth
	(*c*, 0, 0)	−2.134595	−3.653716	−2.957164	−2.617434	Nonstationary
DXNYCK	(*c*, 0, 0)	−3.306002	−3.661645	−2.960415	−2.619160	Smooth
DXNYDK	(*c*, 0, 0)	−1.154629	−3.653716	−2.957146	−2.617412	Nonstationary
	(*c*, 0, 0)	−7.541645	−3.661689	−2.960412	−2.619134	Smooth

**Table 5:** Growth rate of agricultural added value in D county and its proportion in regional GDP.

Years	Agricultural added value (unit: 100 million yuan)	Calculate the growth rate at the price of the current year	Ratio of agricultural added value to regional GDP
2000	1.83	48.00	69.35
2001	2.40	29.73	63.46
2002	3.02	25.83	58.54
2003	3.76	24.5	56.56
2004	5.01	33.24	56.47
2005	6.98	39.46	46.56
2006	9.03	29.35	45.21
2007	11.56	28.59	43.5
2008	15.48	36.16	42.54
2009	17.554	12.26	40.51
2010	19.46	11.28	39.45
2011	22.68	16.59	38.1
2012	26.65	14.16	32.25
2013	29.46	10.54	26.42
2014	31.546	9.46	25.51
2015	36.56	9.46	23.54
2016	37.45	7.54	22.21
2017	38.51	4.56	21.65
2018	39.19	0.56	20.56

## Data Availability

No data were used to support this study.
